# Recommendation of Business Models for Agriculture-Related Platforms Based on Deep Learning

**DOI:** 10.1155/2022/7330078

**Published:** 2022-07-11

**Authors:** Yufei Zhou, Sha Hua

**Affiliations:** School of Business, Hunan Agricultural University, Changsha 410128, China

## Abstract

Agriculture is a basic and pillar industry. With the integration and development of Internet+, platform economy, and various industries, the business model of agriculture-related platforms is also constantly innovating. In this context, it is necessary to recommend suitable business models for different types of agriculture-related platforms. Based on the characteristics of agriculture-related platforms and various business models, this paper proposes a business model recommendation algorithm based on radial basis function neural network (RBFNN). This method trains the RBFNN model with the goal of maximizing the correlation between agricultural-related platforms and business models. In the application stage, for a specific agriculture-related platform, after inputting its characteristic parameters, a suitable business model can be recommended. In the experiment, the proposed method is tested and verified with relevant data, and the results show the effectiveness of the method.

## 1. Introduction

As the consumption revolution triggered by the digital network and the platform economy continues to impact traditional industries, the agriculture-related platforms that combine Internet technology with agriculture have also developed in full swing in the past years [1, 2]. Chinese agriculture is a combination of tradition and modernity. Generally speaking, it is still the type of small farmers in East Asia. It can comprehensively utilize extremely limited resources to the extreme. However, the decentralized agricultural structure is not conducive to the introduction of modern production factors. Also, it is difficult to achieve standardization and large-scale production. How to transform Chinese agriculture from a consumption-based production mode that is overly dependent on resources to a high-quality sustainable green modern production mode is a strategic issue, which needs to be solved urgently in current theoretical research and corporate practice. With the mobile Internet, the large e-commerce companies seriously affected the development of small farmers. However, community group buying cannot fully meet the needs of consumers, and there is a market gap in the production and marketing of agricultural products. However, the development trend of “Internet + agriculture” and agriculture-related platforms is unstoppable. Although agriculture-related platforms are strongly supported by policies, there is still a lack of relevant research on their specific business models.

Early recommendation systems mainly used collaborative filtering (CF) algorithms [3–5]. Subsequently, the recommendation methods based on machine learning algorithms such as support vector machine (SVM) have also been studied and applied [6–8]. In recent years, the deep learning techniques have provided powerful tools for data analysis, and typical models include convolutional neural network (CNN), recurrent neural network (RNN), long short-term memory (LSTM), and so on [9–13]. Relevant applications show that the deep learning methods have superior performance in the field of recommendation algorithms. On the basis of related research, this paper proposes a business model recommendation method for agriculture-related platforms based on radial basis function neural network (RBFNN) [14–16]. The proposed method trains the designed RBFNN with the goal of optimizing the correlation between agricultural-related platforms and business models. On this basis, for the input agriculture-related platform, the best business model can be recommended according to its relevant parameters. The experiments are carried out based on the relevant datasets of agricultural platforms. The results show that the recommendation results of the method in this paper are reliable and have performance advantages compared with several existing methods.

## 2. Background

The business model is the main body and carrier of innovation in the mobile Internet era. It is a complex phenomenon with multiple factors coexisting and intertwined in multiple dimensions, which is a transaction activity to realize a specific value proposition and an important medium for the market and technology. It is widely used in management practice and research and has become a hot research topic in various fields such as organization, strategy, and entrepreneurship. The study of business models begins with the attention to the formation and design of business models. Also, it has gone through many iterations of interpretations by different scholars on the definitions, connotations, and elements of related concepts. First of all, from the definition point of view, the authors in [17] first proposed that a business model is an organic system composed of services, products, and information, which was a unique combination of tangible and intangible assets of an enterprise. Subsequently, the authors in [18] elaborated from the perspective of function, arguing that business model was an important carrier of the ability of enterprises to continuously obtain profits and transformation and upgrading, as well as the key factor to generate enterprise performance. Saebi and Foss [19], through the study of e-commerce model, proposed that a business model was a system of interdependent operational activities between focal enterprises and stakeholders.

In terms of business model innovation, since 2012, some scholars have combined innovation and business model themes and advanced it in depth, which has gradually become the mainstream direction of business model research and has good research and development prospects [20–23]. The innovation of business models is not only an activity of transaction innovation but also a process of institutional innovation and reform in which entrepreneurs and stakeholders interact to create, give, and construct meaning. It is a high-level enterprise innovation behavior including the internal and external factors. It is very different from product innovation, technological innovation, system innovation, and conceptual innovation in the traditional sense. It is a dynamic process of interaction between enterprises and the internal and external environment of the market. Also, there is a changing path that plays a key role in business model innovation. Magretta [20] proposed a method to reconstruct or improve the interaction between the internal components of the business model by redesigning any of the basic elements of the nine elements in its business canvas, such as changing the value proposition of distribution channels and redesigning resource elements. Teece [21] believed that through the innovation or reconstruction of internal elements such as customer segmentation standards, transaction rules, and the relationship between the demander and the supplier, the transformation of the entire transaction system and the innovation of business models can be achieved. Casadesus and Zhu [22] believed that the innovation of internal value drivers and external driving factors can promote the overall innovation of business models.

The research perspective of existing business models mainly starts from the perspective of transaction activities or value creation. The path of business model innovation generally includes element innovation, value proposition innovation, operation model innovation, and business system structure innovation. The authors believe that a business model is the connection transaction method and interest structure between enterprises and stakeholders, which focuses on the value co-creation mechanism of platform business model. The dynamic perspective is mostly based on the value chain, which is difficult to apply to the complex value network created by the platform enterprises through the continuous integration of cross-border resources around the core platform. The static perspective of business model innovation emphasizes the identification and re-emphasis within the business model. It is necessary to construct key elements and core components to realize business model innovation. Also, the research results are too theoretical and not conducive to guiding practice. This research is dedicated to deconstructing and analyzing business model innovation from a systematic perspective, combining static research and dynamic research on business model innovation paths. Therefore, the path of business model innovation is first logically deduced from the perspective of the combination of transaction activities and value creation. By extracting external value drivers and internal attributes, it explains the mechanism and specific change process of the innovation of the platform-based business model of agricultural cooperatives. The core operation logic is that enterprises meet the potential value needs of customers through value proposition innovation, form value maintenance, and ultimately realize the value creation of the entire value network. The constituent units in its framework cover the realization path of business model innovation. Through the design of transaction structure and value creation logic, new value propositions are formed to develop business opportunities and broaden value sources. The platform business is realized through the unique business system structure of value network. Co-creation and sharing of the value of each participant in the ecosystem can increase the added value of consumers' cognitive attachment to products or services. Through the rational allocation of resources, a network effect, scale effect, and monopoly value can be formed. Value co-creation makes economic activities and value transmission change from the one-way path of the traditional value chain to the relationship of value network, which accelerates the efficiency of information dissemination, reduces transaction costs, differentiates products and advantages, and effectively reduces the malicious competition of homogeneous products.

## 3. Method Description

### 3.1. Similarity Model

The business model recommendation problem model involved in this paper includes two entity models: agriculture-related platform and business model. The recommendation problem is actually based on the characteristics of the multiple dimensions of the agriculture-related platform and the business model, to find the minimum difference in the characteristics between the two. Then, a proper way is found to perform accurate matching and to recommend the best business model. Considering the characteristics of agriculture-related platforms and business models, this paper defines the main characteristics of agriculture-related platforms and business models as listed in Table 1.

According to the platform and business model features in the above table, they are first digitally encoded and then we compare the features to find the difference value. Afterwards, the four corresponding feature difference functions *S*_*i*_(*i*=1,2,…, 4) can be obtained, so the recommended model objective function is formed as follows:

(1) $$\begin{array}{c} \min S=\sum_{i=1}^{4}\omega_{i}S_{i}, \end{array}$$

where *ω*_*i*_ represents the weight of different difference functions to the overall recommendation model. According to the recommendation model objective function, for each platform, all available resource features and platform feature differences are sorted in ascending order, and the top-ranked business model is selected to generate a recommendation sequence.

### 3.2. RBFNN

Aiming at the above optimization problem, this paper adopts RBFNN as the basic method to solve it. RBFNN includes a three-layer structure of input layer, hidden layer, and output layer. The relationship between the input layer and the hidden layer is nonlinear, and the relationship between the hidden layer and the output layer is linear. RBFNN uses the radial basis function as the activation function of the neurons in the hidden layer to map an appropriate amount of input to the latent space. Therefore, as long as the center point of the radial basis function is determined, the mapping relationship between the input layer and the hidden layer will also be determined. The hidden layer and the output layer are connected by weights, where the weights are network adjustable parameters. The structure of the RBFNN is shown in Figure 1.

Suppose that the input vector is *X*=[*x*_1_, *x*_2_, ⋯,*x*_*n*_]^*T*^, *n* is the number of input layer units, the output vector is *Y*=[*y*_1_, *y*_2_, ⋯,*y*_*q*_]^*T*^, *q* is the number of output layer units, and the number of hidden layer units is *p*. Here the Gaussian function is used as the kernel function, so the output value of the hidden layer neuron is as follows:

(2) $$\begin{array}{c} h_{j}=\exp\left(-{\left\|\frac{X-C_{j}}{D_{j}}\right\|}^{2}\right),\;j=1,2,\ldots ,p, \end{array}$$

where *C*_*j*_=[*c*_*j*1_, *c*_*j*2_,…,*c*_*jn*_]^*T*^ is the center vector of the hidden layer neuron *j* and *D*_*j*_ is the width vector of the hidden layer neuron *j*, which is related to the action range of the hidden layer neuron on the input; the smaller *D*_*j*_, the narrower the activation function of the neuron *j*; the other neurons have less influence on neuron *j*.

It can be seen from the structure of RBFNN that the input layer and the hidden layer are directly connected, and the hidden layer and the output layer are connected through the weight matrix, which can calculate the initial value of the central parameter, the initial value of the weight, and the width vector. The training process is to solve the network center vector, width vector, and weight matrix of the model.

Figure 2 shows the basic flow of RBFNN training. First, the neural network is initialized. Then, the output results and the root mean square error are calculated with the expected output. If the error meets the termination condition, the training is terminated. Otherwise, the gradient descent method is used to continue to adjust *C*_*j*_, *D*_*j*_, and *W*_*k*_; then, perform cyclic calculation and judge whether the termination condition is met.

### 3.3. Model Realization

According to the above process, the basic process of developing the agricultural platform business model in this paper is described as follows. First, the learning record samples are input. The characteristics of the agricultural platform and business model are encoded and the characteristic variables are input into the RBFNN. The core parameters of the RBFNN are optimized through the algorithms in 3.1 to obtain a stable RBFNN recommendation model. Finally, through multiple training, a stable business model recommendation model for agriculture-related platforms is obtained. The specific condition for iterative stop is whether the feature difference meets the requirements, that is, whether the feature difference reaches the minimum value. According to the trained recommendation model, when a new agriculture-related platform is input, its features can be directly input into the recommendation model, so as to obtain the best business model recommendation result.

## 4. Experiment and Analysis

### 4.1. Dataset

In order to verify the performance of the method in this paper in the recommendation of agricultural platform business model, this section mainly conducts experimental verification. The experimental samples include 4,387 items. Among them, 10 typical business models are included. In the experiment, several types of classic recommendation models in the existing literature are selected as comparison methods, including CF, SVM, and LSTM.

In order to quantitatively evaluate and compare the performance of various methods, the experiments use evaluation indicators widely used in existing literature, including precision (*P*), recall (*R*), and *F*_1_-score (*F*_1_). The definitions of three indexes are as follows:

(3) $$\begin{array}{c} P=\frac{\sum_{u\in U}\left|R\left(u\right)\cap T\left(u\right)\right|}{\sum_{u\in U}\left|R\left(u\right)\right|},\\ P=\frac{\sum_{u\in U}\left|R\left(u\right)\cap T\left(u\right)\right|}{\sum_{u\in U}\left|T\left(u\right)\right|},\\ F_{1}=\frac{2\times P\times R}{P+R}, \end{array}$$

where *R*(*u*) represents the business model selected according to the agricultural platform in the training dataset and *T*(*u*) represents the user's business model recommendation list on the test dataset.

### 4.2. Result and Analysis

Based on the above database, the proposed method and the comparison methods are tested. Also, the statistical results are shown in Table 2. From the results, under the three evaluation indicators, the method in this paper has achieved the best performance, showing its effectiveness. Among the 3 types of comparison methods, the deep learning-based LSTM method has the best performance, reflecting the reliability of the deep learning method in data analysis and prediction. Compared with LSTM, the method in this paper improves the three indicators of *P*, *R*, and *F*_1_ by 2.3%, 2.1%, and 1.7%, respectively, showing the important role of RBFNN in the recommendation algorithm. In conclusion, the method in this paper can be effectively applied to the business model recommendation of agriculture-related platforms and can achieve good results.

## 5. Conclusion

Aiming at the business model recommendation problem of agriculture-related platforms, this paper proposes a recommendation model based on RBFNN. First, the correlation function between agriculture-related platforms and different business models is established, so as to obtain the objective function that needs to be optimized. Then, with the goal of maximizing the objective function, the designed RBFNN is trained to build a recommendation model. For the input agricultural platform, the best business model can be recommended according to its own characteristics. The proposed method is verified by experiments and compared with several existing recommendation algorithms. The results show the effectiveness of the method. By using relevant systems in the development of agriculture-related platforms, it can contribute to the healthy and stable development of agriculture-related platforms.

## Figures and Tables

**Figure 1:** Basic structure of RBFNN.

**Figure 2:** Basic flowchart of RBFNN training.

**Table 1:** Characteristics of agriculture-related platforms and business models.

	Feature	Description
Platform	Content	Specific agricultural areas
	Scale	Funds, personnel, etc.
	Region	Location
	Qualification	Various business qualifications, etc.

Business model	Content category	Agricultural direction involved
	Difficulty level	Requirements for the qualification and scale of the platform
	Popularity	Frequency of use on other platforms
	Region	Applicable regions

**Table 2:** Performance comparison of different methods.

Method	*P*	*R*	*F*_1_
Proposed	0.824	0.873	0.851
CF	0.732	0.758	0.742
SVM	0.727	0.749	0.735
LSTM	0.801	0.852	0.834

## Data Availability

The dataset can be accessed upon request.
